# A Study on the Application Model of Blended Teaching in English Language Teaching in Colleges and Universities under the Ecological and Internet Perspectives

**DOI:** 10.1155/2022/4962753

**Published:** 2022-08-26

**Authors:** Nengsheng Qiu, Xiaoqin Qiu

**Affiliations:** ^1^School of Foreign Languages, Xiamen Institute of Technology, Xiamen 361021, China; ^2^Department of General Education, Xiamen Medical College, Xiamen 361023, China

## Abstract

In order to better adapt to the relevant requirements of blended teaching in colleges and universities under the ecological environment and in the “Internet +” era, the “online + offline” blended teaching mode of college English in the Internet era is innovated to further highlight the subjectivity of students in the process of English learning status. First, this study deeply understands the current situation and problems of College English teaching from the perspective of the Internet by means of a questionnaire survey. On this basis, with the construction of the English teaching concept of “student-centered and teacher-led” as the core, this study puts forward and designs the “online and offline” mixed teaching mode of College English based on the support of mobile network technology. Through the teaching experiment, it is found that the total score of students in the mixed teaching mode is 6 points higher than that before, and the scores for English Cloze, writing, and reading are 2.75 points, 1.3 points, and 1.134 points, respectively. The feasibility and remarkable effect of the mixed teaching mode are verified.

## 1. Introduction

In the context of the rapid development of information technology, blended teaching combines the advantages of traditional teaching and digital teaching to improve the teaching effect. The blended teaching of collegiate oral English under the educational ecological environment builds a mixed classroom ecological environment, provides diverse and open teaching ecological resources for collegiate oral English teaching, and forms a mutually beneficial teacher-student relationship. Today's society has entered the “Internet +” era. Under such a background, the application of electronic information technology and platforms has spread to all walks of life. It can be said that the integration of network and industry provides a strong basic support for the innovation of industrial ecology, and at the same time, it also accelerates the development of education informatization [1]. With the continuous development of the Internet, modern college teaching models are also gradually seeking greater progress. Mu class, micro class, official account learning, and other models have begun to appear. These methods provide more possibilities for further broadening and innovating English teaching methods, which can not only improve students' interest in learning but also further innovate English teaching models. This study is based on this background to deeply explore the innovative development and application of Modern College English mixed teaching mode, and explore the countermeasures and ways more suitable for the innovation of College English teaching mode. Many universities subvert the traditional education mode with the help of Internet thinking and carry out personalized teaching and guidance to students by collecting student data and analyzing and managing these data. In terms of teaching, it adopts the o2o mode across regions and carries out the Internet transformation of the traditional teaching mode into a new way of education. Similar to life in a traditional university, the students in the University also live together and have classes together. The difference is that in the teaching classroom, it is not necessarily the teacher who stands on the podium and gives lectures opposite. It is likely that the teacher stands on the other end of the screen and carries out classroom teaching through webcast interaction [2]. Educational ecology is the concept. Educational ecology is a discipline that uses ecological methods to study the law of human education development. It links education with its ecological environment and analyzes the functions and effects of various ecological factors in the ecosystem. Its interactive relationship with education and human beings aims to create a balanced ecology inside and outside the school, improve teaching efficiency, and seek the direction and countermeasures for the development of the education system.

Gao and others put forward the concept of the flipped classroom, recording the course and uploading it to the Internet for the learning of absent students. Some students return to school after class and ask the teacher to explain in class. Practice has proved that this teaching method has a good effect, so it develops slowly [3]. Flipped classroom can give full play to students' subjective initiative. The most successful case under the flipped classroom teaching mode is the teaching mode of Khan college. Browsing the videos on the Khan Academy website, you will find that they have no fancy pictures, no eloquent teachers, only a blackboard and Mr. Khan's narration. All this is to lead the students to think and learn synchronously with the video course. The next goal of Khan college is to prepare most courses from kindergarten to university and translate them into multiple languages. In terms of academic research, the Ministry of education and major key universities have launched a series of online courses. However, in the actual process of education and teaching, due to the lack of structural reform of education model, online course teaching is not used in the teaching process at a deeper level [4, 5]. At the same time, with the expansion of network construction from large and medium-sized cities across the country to urban areas and remote rural areas, the expansion and teaching use of network courses have high promotion potential and value. The teaching research of network courses can be summarized as follows:

Personalized learning: the future learning of online courses can well arrange the learning progress of online courses, take students as the center, teach students according to their aptitude, and meet their personalized learning resources and learning methods. Through the test of students' learning ability and course mastery level, intelligently recommend the courses required by students.

Shared learning resources: it is necessary to establish a distributed shared learning platform and improve the resource sharing of network resources among colleges and universities by combining the advantages of centralized and local deployment of network courses. This also requires that the design of network courses follow the basic unified standards and can realize the identity authentication of user registration and the big data analysis and management of network courses.

Virtual laboratory: the learning of online course only shows the experimental process, data and results to students, but can not let students immerse themselves and participate in the experiment of the course. Virtual laboratories can let students reflect on the experimental process and observe the experimental results and phenomena through virtual reality technology.

## 2. Investigation on the Current Situation of Online Course Teaching in Colleges and Universities from the Perspective of Internet

### 2.1. Investigation Purpose and Method

#### 2.1.1. Purpose

Take college students as the research object, investigate and understand the current situation of network curriculum education in Colleges and universities, analyze the individual differences and existing problems of network curriculum teaching, and students' suggestions for network curriculum.

#### 2.1.2. Method

A questionnaire survey was conducted on students in local colleges and universities, and the data were analyzed by SPSS, so as to provide data reference for the research of online and offline hybrid teaching mode for college students. Through the class cluster sampling method, the college students of a university English college are selected as the sample and tested under unified guidance [6]. A total of 550 questionnaires were distributed and 503 valid questionnaires were recovered, with an effective rate of 91.5%. See Table 1 for the basic information of the respondents, including 347 boys, accounting for 70.1% and 134 girls, accounting for 27.7%; 261 freshmen, accounting for 52.8%, and 212 sophomores, accounting for 45.1%.

In online course learning, students study independently online, complete the course content and chapter tests, and achieve their learning objectives through the functions and services of the platform, such as Q&A, discussion, resources, and so on. The assessment of learning quality generally includes three parts: video viewing (40%), usual homework (20%), and final examination score (40%). At present, online courses have a course forum module, through which students can ask questions about knowledge points and other related courses, get the help of teachers and teaching assistants, and have joint discussions among students [7].

The questionnaire is designed according to the psychological factors that affect the learning effect of online courses and combined with the characteristics of English learning. There are 34 questions in this questionnaire, 2 basic personal information, and 31 main survey questions. The main part is divided into six dimensions: 1. The degree of understanding of online courses (4); 2. Classroom participation (5 channels); 3. Satisfaction with teaching (5); 4. Technology application (3 channels); 5. Sense of harvest (7 channels); 6. Constructive suggestions (6). It includes single-choice questions and open-ended questions. There are 24 single-choice questions in the first five dimensions, which mainly adopt the four-level scoring standard. The higher the score, the better the teaching effect of online courses; The sixth dimension includes choice and open-ended questions. There are 6 questions in total, which are not scored. The data were analyzed by SPSS18.0. The data show that the questionnaire has good reliability and validity and can be used as an evaluation tool for the current situation of College Students' Online Course Teaching [8, 9].

### 2.2. Results and Analysis

#### 2.2.1. Data Statistics and Analysis

Descriptive statistics were made on the subjects' understanding, classroom participation, satisfaction, technology application and sense of harvest. The results are shown in Table 2. The survey data show that the total score of College Students' current situation of online course teaching (42.64 ± 13.50), degree of understanding (6.84 ± 2.56), classroom participation (9.86 ± 3.39), satisfaction (8.35 ± 2.96), technology application (5.29 ± 1.96) and sense of harvest (12.31 ± 4.73). The average value of a single item (1.67), the average value of awareness (1.60), the average class participation rate (1.86), the average satisfaction (1.56), the average technology application (1.65), and the average value of sense of harvest (1.65) of the current situation of online course teaching of College students are less than the theoretical median value of a single item (2.5) [10]. It can be seen that the current situation of College Students' online course teaching needs to be improved. There are individual differences in the current situation of College Students' online course teaching, but it needs to be improved in terms of consciousness, classroom participation, satisfaction, technology application, and sense of harvest.

As can be seen from Table 3, the first three scores of a single item are B5 (2.17) and B2 (2.17). Among the other 21 items, the scores are between 1.47 and 1.97, with the largest SD item being 1.3 and the smallest SD item being 0.55 for the B4 item.

In terms of College Students' understanding of the current situation of online course teaching, there are four topics to evaluate the knowledge understanding. The overall students' knowledge dimension score is 6.84 (Full Score 16), and the average score of each item is 1.71 (theoretical median is 2.5). This shows that students' understanding of the current situation of network course teaching is not enough.

In terms of classroom participation in the current situation of College Students' online course teaching, there are five topics to evaluate the knowledge understanding. The overall students' knowledge dimension score is 9.86 (out of 20 points), and the average single score is 1.97 (the theoretical median is 2.5). This shows that the current situation of students' participation in online course teaching in class is not enough.

From the aspect of satisfaction with the current situation of College Students' online course teaching, there are five topics to evaluate the knowledge understanding. The overall students' knowledge dimension score is 8.35 (full score is 18 points), and the average score of each item is 1.67 (theoretical median is 2.5 points). This shows that students' satisfaction with online teaching is not enough.

In terms of the technical application of the current situation of College Students' online course teaching, there are three topics to evaluate the knowledge understanding. The overall students' knowledge dimension score is 5.29 (out of 12 points), and the individual average score is 1.76 (the theoretical median is 2.5). This shows that the technical application of students' network course teaching is not enough.

In terms of the sense of harvest of the current situation of College Students' online course teaching, there are seven topics to evaluate the knowledge understanding. The overall students' knowledge dimension score is 12.31 (out of 28 points), and the average single score is 1.76 (the theoretical median is 2.5). This shows that students' online teaching is not enough [11, 12].

The comparison of gender differences in the current situation of online course teaching is shown in Table 4. The *t*-test results show that the total score, classroom participation, technology application and sense of harvest of boys are significantly lower than those of girls (*P* < 0.01), and the two dimensions of boys' awareness and satisfaction with the Internet are significantly lower than those of girls (*P* < 0.05).

In the sixth dimension, in terms of constructive suggestions on the current situation of College Students' online course teaching, this study has six topics to evaluate understanding of knowledge. When asked about the courses that college students think online courses are suitable, as shown in Figure 1.

When asked about the links that college students think are suitable for online courses (as shown in Figure 2), the number of preclass previews, postclass reviews, teacher-student communication, and others are 196, 143, 131, and 33, respectively, accounting for 39%, 28%, 26%, and 7%, respectively, which shows that college students think that preclass preview is suitable for online course teaching, but not for online teaching in terms of teacher-student communication.

When asked which type of resources college students prefer teachers to provide (as shown in Figure 3), the number of reference books, courseware/lesson plans, videos, learning websites, and others are 117, 117, 213, 52, and 4 respectively, accounting for 23%, 23%, 42%, 10%, and 1%, respectively, which shows that college students think they prefer video resources rather than teachers to provide learning website resources.

When asked about the appropriate length of time for college students to adopt network teaching for a course (as shown in Figure 4), the number of people within 1 hour, 1-2 hours, 2-3 hours, and more than 3 hours are 304, 155, 30 and 14, respectively, accounting for 60%, 31%, 6%, and 3%, respectively, indicating that college students think the appropriate length of time for a course to adopt network teaching is within 1 hour.

Based on the above survey results, colleges and universities need to fully tap and make use of their rich educational resources according to the actual situation of schools and students, and promote the integration of online course teaching and traditional teaching forms, that is, hybrid teaching based on online courses [13–15].

### 2.3. The Characteristics of the Blended Teaching of Collegiate Oral English under the Ecological Environment

The construction of the ecological system of the mixed teaching of collegiate oral English in the ecological environment includes three ecological factors: “teachers,” “students” and “teaching ecological environment.” The three ecological factors of teachers, students and teaching ecological environment have different connotations. The three are interdependent and interact with each other, and they are an organic part of the college English teaching ecosystem. From the perspective of the ecological environment and teaching ecological resources, the author analyzes the ecological characteristics of college English mixed oral teaching.

#### 2.3.1. Hybrid Classroom Ecological Environment

In the past, traditional college English classrooms were still relatively simple. Teachers input a large amount of corpus through face-to-face teaching and interaction in the classroom, providing students with a face-to-face communication and interaction platform for oral expression and output, and urging students to internalize the input into oral expression ability. However, due to the limited class hours of college English classes and the large number of students, the teaching effect is reduced. And the effect of oral English teaching is not only related to teachers' classroom teaching, but also proportional to the amount of students' oral language training. In view of the lack of oral practice in face-to-face classrooms, online teaching can provide students with massive learning resources and a variety of real-time communication tools, breaking through time and space constraints and meeting the requirements of learning and practicing anytime, anywhere. Under the guidance of teachers, students can use various online teaching platforms to complete oral practice tasks individually or in groups. Teachers conduct detailed assessments of students' oral language training through the online teaching platform, and can also use QQ, WeChat and other social software to answer questions and guide online promptly, supplement the interaction with students, and effectively meet the needs of students for independent learning after class. Students can use the fragmented time after class to realize oral practice anytime and anywhere, so as to make up for the shortcoming of the lack of classroom oral practice time. The hybrid construction of the traditional college oral English classroom and the online classroom fully combines the advantages of the two, complementing and complementing each other, greatly improving the teaching efficiency.

#### 2.3.2. Diverse and Open Teaching Ecological Resources

In the era of rapid knowledge update, the traditional paper-based college oral English teaching materials often have a certain lag, and the subject matter lacks modernity and novelty, which reduces students' interest and enthusiasm for learning. In addition, the limited teaching resources of textbooks make it inconvenient for students to carry out independent study after class. In the Internet + era, it is very convenient to obtain massive resources. These learning resources have a wide range of topics, various forms, and strong timeliness. These pure and authentic learning resources allow students to directly input real spoken language materials, and also understand cultural customs and cultural differences, which is conducive to stimulating their interest in learning and arousing their enthusiasm for learning. In college oral English teaching supported by information technology, teachers can either directly click on network links in the classroom teaching environment to share online learning resources with students, or use other online learning platforms and other resources to organize teaching. Therefore, under the blended teaching mode, the teaching resources of college oral English teaching not only include traditional learning resources such as textbooks, but also various mobile learning software, MOOCs and other learning platforms, and micro-courses, and other fragmented resources. Teachers can use micro-courses, MOOCs, and other teaching methods to improve the efficiency of classroom teaching, arrange students to conduct independent learning, and check and fill vacancies. Teachers can also use various online teaching platforms to supervise and detect voice and video resources such as voice exercises, dialogue exercises, and group activities completed by students, and can also easily forward outstanding students' works to achieve resource sharing. After class, teachers can use social software such as WeChat group and QQ group, or teaching platforms such as Xuetong to release learning resources such as courseware and exercises to students, and supervise students' after-school exercises through the teaching platform.

## 3. Correlation Analysis of College Students' English Mixed Teaching Mode Supported by Mobile Network Technology

The teaching experiment course is an elective second foreign language English course for non-English majors. The teaching material is New Horizon College English. According to the time sequence of students' course selection, the teaching management system randomly arranges the course selection students into four classes. Two classes are selected, one of which is the experimental class for mixed teaching experiments; The other class serves as the control class. In addition to normal teaching, the teachers in the control class do not intervene outside the classroom. For the experimental class, the mixed teaching experiment is designed and implemented according to the “target oriented mixed teaching model.” Before class, mobile devices are used for collaborative learning, independent exploration, activities, testing, and evaluation. In class, mobile devices are used to optimize teaching methods, and a mixed teaching experiment supported by mobile technology with target as the guide, communication and interaction as the core, and forming “teacher leading student subject” is established [16].

### 3.1. Analysis of Influencing Factors

In recent years, the acceptance model of mobile learning mainly draws lessons from the “UTAUT model” formed by integrating eight technical theoretical models such as innovation diffusion theory. The model is shown in Figure 5.

Referring to the UTAUT model and combined with practice, the author constructs a research framework on the influencing factors of College Students' acceptance of English mobile learning (Figure 6). Referring to the existing scale, formulate a questionnaire and analyze the influencing factors of College Students' acceptance of mobile learning English through the questionnaire [17–19].

### 3.2. Research Scheme

Develop a questionnaire. The questionnaire adopts Likert's five-level scale, which expresses the degree of recognition of the respondents from the five levels of “very inconsistent,” “relatively inconsistent,” “uncertain,” “relatively consistent” and “very consistent,” and the corresponding score is 1–5. The respondents are students of three grades in a university, without professional restrictions. This study uses campus app software to send questionnaires to students and collect questionnaires. A total of 894 questionnaires were collected and 49 were invalid, with an effective rate of 94.5%. Demographic variables are shown in Table 5.

The data analysis of the questionnaire is processed in Excel software and the data analysis of the questionnaire is processed by Excel software and spss220 software. On the premise of complying with the research norms, descriptive statistics, reliability and validity test, regression analysis, difference test, and other analysis methods are carried out on the overall data and dimensions of the questionnaire [20].

### 3.3. Data Analysis

The analysis results show that (see Table 6), the overall reliability of the questionnaire is Cronbach' *a* = 0.851, and the coefficient of each variable of the scale is basically about 0.8, indicating that the questionnaire has good reliability. The validity of the scale was tested. The results showed that KMO = 0.970 > 0.8, Bartlett's spherical test *p* ≤ 0.01, indicating that the scale is suitable for factor analysis. Through the exploratory factor analysis of the questionnaire by the method of principal component analysis, the variance interpretation rate of the six factors is 66.329%, which is greater than 60%, indicating that the structural validity of the scale is good. software.

After questionnaire survey and data analysis, the following conclusions can be drawn from the research on the influencing factors of mobile learning:

1. There is a significant positive correlation between the five factors selected in the study.
2. The adjustment variables have significant differences in the adjustment of various influencing factors. Female students are more receptive to mobile learning than male students, and senior students pay more attention to the richness and quality of English mobile learning content and resources.
3. Perceived self-efficacy, content, resources, and performance expectations are the key factors affecting college students' English mobile learning behavior intention.

### 3.4. Implementation Cases of Mixed Teaching

Students are at CET-4 level, and the other half fail to pass CET-4. Vocabulary is the basis for learning and mastering a language. Therefore, students' mastery of vocabulary is emphasized in teaching. According to the textbook, the new unit requires students to focus on learning 8 phrases in this unit and basically master 21 words. It is required that the keywords to be mastered should be subject to targeted training, be able to choose, match and use words, and be able to understand and remember the basic words. Before the formal course, release learning objectives, upload learning contents and resources to students through the online platform, and organize the discussion. The learning objectives of students' autonomous learning stage: recognize and memorize the words required by the new unit and complete the after-school exercises of the previous class [21, 22].

In order to enable students to better understand and memorize new knowledge, the text recording of unit 4, the PPT and recording of vocabulary and example sentences required to be basically mastered, the single choice questions of relevant vocabulary and upload them to the classroom before class. Students are required to learn the uploaded PPT and recording of the new class within the specified time while completing online after-class exercises, complete the vocabulary test, and publishing the recording of personal new words in the discussion area. Teachers organize online discussions, communicate with teachers and students, and share key pronunciation points, difficult words, etc. In class, the main teaching task is to explain the key phrases based on making students understand the basic words. The teacher uploads the courseware to the classroom to send teachers and students to the same screen and sets interactive answers at the key knowledge points required in the courseware. Under the condition that teachers and students are on the same screen, students can synchronize the courseware with teachers through a mobile phone applet, so as to avoid problems such as old projection equipment, unclear projection, and unclear courseware content; Students can also send real-time bullet screens, and questions generated in class can be raised through bullet screens; When the teacher teaches key phrases, click the interactive answer button, and the students can receive a message reminder through the mobile phone. Click to participate in the answer. After completing the answer within the time limit, the students' answer can be displayed on the teacher side. Through this interactive way, teachers can improve students' interest in learning, improve students' classroom participation, and promote one to many communication between teachers and students in the classroom in a sense. On the other hand, it can help teachers examine the mastery of each student's new knowledge. At the end of the class, the teacher assigns homework: according to the newly learned words/phrases, students choose 3–5 as the core words/phrases, write a composition of about 120 words on the correction website, and complete it within the time limit.

## 4. Experimental Analysis of the Mixed Teaching Mode

### 4.1. Experimental Design

The teaching experiment takes half a semester as the experimental cycle, and the formal teaching time is from the ninth week to the sixteenth week. The experimental hypothesis is that the hybrid teaching of College English courses supported by mobile technology can improve college students' English listening and speaking ability, reading ability, writing and translation ability, and comprehensively improve college students' English learning effect. Select two classes, one class as the experimental class, and carry out the mixed teaching experiment; The other class serves as the control class. In addition to normal teaching, the teachers in the control class do not intervene outside the classroom. After considering the demographic variables such as the total number of classes and gender, class C is selected as the intention control class. The author uses the test paper formulated according to the unified standard of the school in the previous academic year as the test question before the experiment of this period. The test time is limited to 180 minutes. The test content includes six major questions, with a total score of 100 points. The test results show that there is no significant difference in the scores and total scores of the six major questions, and the experimental class is homogeneous with the control class C. Therefore, class C is finally determined as the control class of this experiment.  Table 7 shows the comparison of the results before the experiment between the experimental class and the control class.

Considering that other variables other than experimental variables may affect the teaching experiment results, in order to reduce the impact as much as possible, the author controls the additional relevant variables:

1. Teachers are constant. The author contacted an English teacher in a university, showed the teacher the purpose of the experiment, and reached a teaching experiment cooperation with him. In order to avoid the influence of different teachers in the experimental process on the experimental results, the experimental class and the control class are selected from the class taught by the teacher to ensure that the teachers are constant;
2. The class is random. The teacher undertakes four classes of English courses, from which class D is selected as the experimental class; The English classes in the experimental class are scattered on Monday and Friday, and other courses are concentrated on Monday, Tuesday, and Thursday. There are no evening courses and weekend courses except Tuesday. Therefore, the students in the experimental class have sufficient time for autonomous learning and group cooperative learning. Every student in the experimental class has a smartphone that supports Internet access, video playback, recording, file access, and other functions. 90% of the students are equipped with laptop computers, and about 80% of the students have Walkman (MP3/4/5), learning machine or tablet computer and other devices that can support mobile learning, which meet the necessary conditions of hybrid teaching experiment.

### 4.2. Experimental Data Benign Research

Experimental difference analysis. Paired sample *t*-test was used to analyze the pretest and posttest results of the experimental class. According to the analysis results (Table 8), there are significant differences in the total score, cloze test, Chinese-English translation and writing of the pretest and posttest scores of the experimental class, and the average scores of the posttest in the total score, cloze test, Chinese-English translation and writing of the experimental class are greater than the average scores of the pretest, indicating that the students have significantly improved in these four aspects. Among them, the difference level of “Chinese-English translation” is *P* < 0.05, the difference level of “cloze test” is *P* < 0.01, and the difference level of “total score” and “writing” is the highest, *P* < 0.001.

## 5. Conclusion

Based on certain teaching objectives, hybrid teaching organically integrates traditional classroom teaching with modern network learning, and organically integrates a variety of teaching elements, so as to optimize the teaching effect. In mixed teaching, teachers can maximize their play as guides, learners as teaching subjects, give full play to their creativity and imagination in cooperative exploration, and get personalized development in autonomous learning. This paper proposes and designs a “online and offline” mixed teaching mode of College English based on mobile network technology. Through the analysis of the teaching experimental results, we can draw the following conclusions:

1. The hybrid teaching mode supported by mobile technology can improve students' reading ability, writing and translation ability; When the experimental period is not long, the total score of the students in the experimental class is 6 points higher than that in the pretest, and the scores of cloze, writing and reading in the posttest are 2.75 points, 1.3 points and 1.134 points higher than that in the pretest. The total scores of the control class are not significantly improved in the posttest and pretest, but only the writing score is increased by 0.867 points. From this, it can be seen that the performance of the experimental class is significantly improved, and the effect of the mixed teaching mode is remarkable.
2. Through the mixed teaching mode, college students' English learning effect is comprehensively improved; This study constructs a hybrid teaching model supported by mobile technology by using the goal-oriented teaching model, which improves the teaching effect and students' performance significantly. Combined with quantitative analysis, formative evaluation and teacher feedback, we can know that under the mixed teaching mode, students have strong learning interest and learning atmosphere, and their learning initiative has been enhanced. Through group activities and online discussion, students' listening and oral pronunciation have been improved, and students have gradually established English self-confidence in the whole process.
3. Due to the unified proposition test paper, the experimental research can not conduct quantitative analysis on listening and speaking, and can not use the data to clearly judge whether the students in the experimental class have significantly improved in listening and speaking, which can only be judged by the supervisor of the teacher.

## Figures and Tables

**Figure 1:** Courses that college students think e-learning is suitable for.

**Figure 2:** Links that college students think online courses are applicable.

**Figure 3:** What kind of resources do college students prefer teachers to provide?

**Figure 4:** The appropriate length of time for college students to adopt network teaching in a course.

**Figure 5:** UTAUT model.

**Figure 6:** Research framework.

**Table 1:** Basic information of respondents.

Item	Option	Number of people	Percentage
Gender	Male	347	70.1
	Female	134	27.7
Grade	Freshman	261	52.8
	Sophomore	212	45.1

**Table 2:** Descriptive statistics of each dimension score of college students' online course teaching status.

Category	Score range	*M*	SD	Single mean
A degree of awareness	4–16	6.73	2.45	1.60
B classroom participation	5–20	9.75	3.28	4.86
C satisfaction	5–18	8.24	2.85	1.56
D technology application	3–12	5.18	1.85	1.65
E sense of harvest	7–28	11.21	4.62	1.65
Total score	24–88	41.56	12.40	1.67

Note: *M* refers to the average value and SD refers to the standard deviation.

**Table 3:** Description and statistics of the current situation of online course teaching for college students.

Item	*M*	SD
A1	1.51	0.62
A2	1.70	0.76
A3	1.57	0.68
A4	1.62	0.71
B1	1.86	0.75
B2	2.07	0.88
B3	1.85	0.61
B4	1.36	0.55
B5	2.17	1.00
C1	1.61	0.61
C2	1.53	0.61
C3	1.58	0.61

**Table 4:** Gender differences in the current situation of online course teaching.

	Male (*n* = 347)		Female (*n* = 134)		*T*
	*M*	SD	*M*	SD	
Degree of understanding	5.55	2.46	7.17	2.37	−2.405^*∗*^
Classroom participation	9.35	3.31	10.73	3.01	−4.277^*∗*^
Satisfaction	8.07	2.87	8.66	2.80	−2.045^*∗*^
Technology application	5.01	1.80	5.61	2.04	−2.010
Sense of harvest	10.60	4.46	12.70	3.70	−3.385^*∗*^
Total score	40.01	12.33	45.31	11.82	−3.006^*∗∗*^

Note: ^*∗*^, *P* < 0.05; ^*∗∗*^, *P* < 0.01.

**Table 5:** Demographic variable information.

External variable		Frequency	Percentage
Grade	Grade 2017	157	18.8
	Grade 2018	306	36.4
	Grade 2019	350	41.5

Gender	Male	410	48.7
	Female	423	50.1

Professional category	Liberal arts	270	32.2
	Science	553	65.6

**Table 6:** Analysis of variables and reliability.

Variable	Cronbachs alpha	Number of items
Holistic scale	0.851	29
Performance expectation	0.686	4
Effort expectation	687	4
Social influence	0.712	4
Perceived self energy efficiency	0.678	4
Content and resources	0.718	4
Behavioral intention	0.714	4

**Table 7:** Comparative analysis of results of experimental class and control class before experiment.

Item	Compared with the results of preclass test		Pretest results of experimental class		*t*
	Average	Standard deviation	Average	Standard deviation	
Total score	78.256	8.556	77.572	7.410	0.215
Banked cloze	13.456	10.012	13.072	2.260	1.052
Cloze test	7.100	3.161	8.540	2.722	−0.414
Reading comprehension	13.500	2.682	12.422	2.737	1.070
English Chinese translation	8.60	0.823	8.700	0.251	−0.436
Chinese-english translation	8.400	1.071	8.315	0.827	0.2180
Writing	21.800	2.122	22156	1.373	−0.938

Note: ^*∗*^, *P* < 0.05, ^*∗∗*^, *P* < 0.01, and ^*∗∗∗*^, *P* < 0.001.

**Table 8:** Analysis on the difference of scores before and after the experimental class.

Item	Pretest scores of control class		Pretest results of experimental class		*t*
	Average	Standard deviation	Average	Standard deviation	
Total score	77.572	6.410	83.616	5.887	−3.120^*∗∗∗*^
Banked cloze	13.072	2.161	13.356	0.770	−0.705
Cloze test	8.640	3.722	10.300	3.476	−3.108^*∗∗*^
Reading comprehension	12.422	3.737	13.556	3.551	−1.484
English Chinese translation	8.700	0.251	8.700	0.226	0.001
Chinese-English translation	8.316	0.827	8.740	0.187	−2.402^*∗*^
Writing	22.156	1.373	23.456	1.005	−3.881^*∗∗∗*^

Note: ^*∗*^, *P* < 0.05, ^*∗∗*^, *P* < 0.01, and ^*∗∗∗*^, *P* < 0.001.

## Data Availability

The labeled data set used to support the findings of this study is available from the corresponding author upon request.
